The article "Mechanism of Anti-Inflammatory Drugs in the Early Treatment of Oral Gingival Mucosa and Soft Tissue Trauma" was retracted in 2023. Reasons: signs of a paper mill; compromised peer review; unreliable results or conclusions.

# Mechanism of Anti-Inflammatory Drugs in the Early Treatment of Oral Gingival Mucosa and Soft Tissue Trauma

**DOI:** 10.1155/2022/5785025

**Published:** 2022-09-29

**Authors:** Yanfeng Zhu, Fei Lin, Weihui Chen

**Affiliations:** Department of stomatology, The Affiliated Union Hospital, Fujian Medical University, Fuzhou 350001, Fujian, China

## Abstract

Traumatic tissue develops an uncontrolled inflammatory response that causes secondary damage to the injured tissue and other parts of the body. Therefore, preventing wound infection, reducing inflammatory response, and reducing secondary tissue damage are the keys to early treatment of tissue trauma. In the treatment of gingival soft tissue trauma, anti-inflammatory and analgesic drugs are reasonably selected according to the condition, which can effectively reduce inflammation, and they help periodontal tissue regeneration and healing. However, there are few studies on the mechanism of anti-inflammatory drugs in the early treatment of oral gingival mucosal soft tissue trauma, and the specific mechanism is unknown. Therefore, this paper explored the mechanism of anti-inflammatory drugs in the early treatment of oral gingival mucosa and soft tissue trauma through experiments, which provided theoretical support for the clinical treatment of gingival mucosa and soft tissue trauma repair. In this paper, two anti-inflammatory drugs, levofloxacin and metronidazole, were selected to measure their release properties *in vitro* and *in vivo*. Then, the white-eared rabbits were treated with gingival wound treatment experiments, and the physiological characteristics, intratissue pressure, tissue partial pressure of oxygen, IL-6 content, and PGE2 content were determined at each postinjury period, and the mechanism of action of anti-inflammatory drugs was determined. Research results have shown that anti-inflammatory drugs can significantly inhibit the content of IL-6 and PGE2 in gingival soft tissue after injury, reduce the local inflammatory response, and accelerate tissue healing.

## 1. Introduction

Gum soft tissue trauma is common in dentistry for several reasons: the gums are clamped when forceps are placed; the gums are not completely separated during extractions and remain attached to the teeth, causing tearing; other reasons, such as the extraction of maxillary wisdom teeth, are often caused by excessive force when levering the tappet distally, which may cause tearing of the attached gingiva on the buccal and palatal sides of the wisdom teeth; twisting the soft tissue when using a turbodrill can cause varying degrees of soft tissue trauma. At present, gingival soft tissue trauma is often treated with anti-inflammatory drugs in the early stage, which can effectively organize the inflammatory response caused by trauma and have a very good curative effect. However, at present, there are few studies on the mechanism of anti-inflammatory drugs in the early treatment of gingival mucosa and soft tissue trauma, so further research is still needed.

The article "Mechanism of Anti-Inflammatory Drugs in the Early Treatment of Oral Gingival Mucosa and Soft Tissue Trauma" was retracted in 2023. Reasons: signs of a paper mill; compromised peer review; unreliable results or conclusions.

At present, there are many studies on soft tissue trauma. Vajs et al. described the clinical presentation, diagnostic procedures, management (emphasis on type, duration, and route of antimicrobial administration), and outcomes in cases of acute soft tissue trauma to the tarsal region. He assessed clinical features, outcomes of diagnostic modalities, and initial response to therapy to determine their usefulness in predicting SI [1]. Matei et al. conducted a one-year retrospective case-control study at two hospitals to evaluate soft tissue trauma after vaginal delivery in adolescent mothers compared with adult mothers [2]. Hampp et al. compared the extent of soft tissue trauma maintained by robotic arm-assisted PKA and manual PKA in knee arthroplasty [3]. Ko et al. reviewed the current literature involving soft tissue trauma to the eyelid and periorbital tissue and highlighted key steps in the evaluation and management of patients with various types of injuries [4]. Houle et al. outlined the goals of managing lip soft-tissue trauma, as well as the appropriate examination and eventual treatment of various types of lip soft-tissue trauma [5]. Although there are more studies on soft tissue trauma, there are fewer studies on gingival mucosal soft tissue trauma.

Many scholars have studied the mechanism of action of anti-inflammatory drugs. Boakye et al. studied the potential molecular target of Trichoderma, and the results showed that the anti-inflammatory mechanism of Trichoderma leads to the inhibition of NF-*κ*B and the increase of Nrf2 activity [6]. Li et al. studied the anti-inflammatory mechanism of water-soluble Ginkgo biloba polysaccharides through bioinformatics analysis. The specific mechanism may be related to its regulation of the expression of p-p65, p-I*κ*B*α*, TNF-*α,* and IL-1*β* proteins in the inflammatory signaling pathway [7]. Abdelghany et al. investigated the possible anti-inflammatory effects of nicaraven in slowing tumor growth. Studies have shown that nicaraven can effectively prevent the rapid growth of inflamed tumors through anti-inflammatory mechanisms [8]. Zhang et al. studied the anti-inflammatory mechanism of Polygonum vulgaris through network pharmacology and obtained 11 active ingredients and 183 protein targets through screening [9]. Olubanke et al. studied the anti-inflammatory activity of ORuzu herbal bitter (RHB) and confirmed the anti-inflammatory activity of RHB in the prevention of NAFLD in rats [10]. Although there are many studies on the mechanism of action of anti-inflammatory drugs, there are few studies on the early treatment mechanism of anti-inflammatory drugs on oral gingival mucosa and soft tissue trauma.

The article "Mechanism of Anti-Inflammatory Drugs in the Early Treatment of Oral Gingival Mucosa and Soft Tissue Trauma" was retracted in 2023. Reasons: signs of a paper mill; compromised peer review; unreliable results or conclusions.

In this paper, the anti-inflammatory drugs for the early treatment mechanism of oral gingival mucosa and soft tissue trauma were studied. In this study, two anti-inflammatory drugs, levofloxacin and metronidazole, were selected. First, the release properties of the drug *in vitro* and in vivo were measured, including the release experiment of the drug *in vitro* and the distribution of the drug in the body to explore the drug release properties. Then, the role of anti-inflammatory drugs in the early management of gingival mucosa and soft tissue trauma was studied, including the determination of wound healing, body temperature, respiratory rate, heart rate, pressure in wound tissue, partial pressure of oxygen in wound tissue, IL-6 content, and PGE2 content in wound tissue after gingival trauma in animals to determine the mechanism of anti-inflammatory drugs in the early management of gingival mucosa and soft tissue trauma.

## 2. Experimental Materials, Reagents, and Instruments

### 2.1. Experimental Materials

Eighteen 4-month-old male big-eared white rabbits were purchased from the Hubei Provincial Laboratory Animal Research Center.

### 2.2. Experimental Drugs and Reagents

Levofloxacin Tablets (Xinchang, Zhejiang), Metronidazole Tablets (Xifeng, Liaoning), Interleukin 6 (IL-6) Kit (Shanghai Blue Base), and Prostaglandin E2 (PGE2) Kit (Nanjing Jiancheng) were used.

Acetonitrile, sodium citrate, triethylamine, sodium acetate, phosphoric acid (Sinopharm Group) were also used.

### 2.3. Experimental Equipment

SPD-10A.VP Shimadzu high-performance liquid chromatograph (Japan); MettlerAE200 dual-range analytical balance (Shanghai); SK320 type 100 kg piezoresistive sensor (Yangzhou, Jiangsu); LicoxLPM tissue oxygen partial pressure monitor (Germany); Glass tissue grinder (Chongqing); Sartorius electronic balance (Japan).

## 3. Determination of Release Properties of Anti-Inflammatory Drugs *In Vitro* and *In Vivo*

### 3.1. Drug Release Experiment *In Vitro*

Three levofloxacin tablets and three metronidazole tablets were selected, 900 ml of normal saline was used as the solvent, and the temperature of the solvent was kept at about 37°C by heating. The soaking water was replaced at each point of 4 h, 8 h, 12 h, 16 h, 20 h, and 24 h, and 10 ml of the soaking liquid was taken at each time point. After filtration, 2 ml was accurately measured and placed in a 100 ml volumetric flask. 0.1% mol/L hydrochloric acid solution was diluted to the mark and added and shaken. The absorbance of levofloxacin was measured at a wavelength of 293 nm, and the absorbance of metronidazole was measured at a wavelength of 277 nm by high-performance liquid chromatography [11]. The cumulative dissolution percentage *S*% is calculated according to the following formula:

(1) $$\begin{array}{c} S\%=A_{i}A_{0}>100\%,\\ A_{0}=W_{0}W_{m}. \end{array}$$

Among them, *A*_*i*_ is the absorbance, and *A*_0_ is the absorbance of all the tablets dissolved. *W*_*m*_ is the average sheet weight, and *W*_0_ is the corresponding weight of each sheet.

The article "Mechanism of Anti-Inflammatory Drugs in the Early Treatment of Oral Gingival Mucosa and Soft Tissue Trauma" was retracted in 2023. Reasons: signs of a paper mill; compromised peer review; unreliable results or conclusions.

### 3.2. Determination of Drug Distribution *In Vivo*

#### 3.2.1. Sample Collection

There were 6 big-eared white rabbits. For each sample, the maxillary and mandibular gingiva was used as research objects, and the labial gingiva was excised 2 mm with a scalpel. Debridement was performed after injury, and 1 capsule was administered. Each animal was injected with 50 ml of 0.9% NaCl solution, and the animals were allowed to eat and drink ad libitum. At 6 h, 12 h, 24 h, and 36 h after injury, 1 ml of venous blood was drawn and stored in a −30°C refrigerator; about 0.1 g of muscle tissue was taken 1.5 cm away from the wound and stored in a −30°C refrigerator [12].

#### 3.2.2. Sample Processing

The cryopreserved blood sample was taken out, and after centrifugation, 0.5 ml of the supernatant was taken, and 0.6 ml of 1 mol/L phosphoric acid solution was added. After mixing, 5.0 ml of an extract prepared with n-hexane and isopropanol was added, and the volume ratio of the extract was 95:5. Extracted with a vortex mixer for 2 min and centrifuged for 10 min (3000 r/s), 4 ml of the upper organic liquid was extracted and air-dried at 40°C. The residue was completely dissolved in 150 *μ*l of the mobile phase. It was centrifuged again at 3000 r/s for 10 min, and 25 *μ*l of the supernatant was taken for injection and determination by a high-performance liquid method [13].

Cryopreserved tissue samples are removed and accurately weighed. It was placed in a vial with 2 ml of normal saline, minced, and homogenized with a tissue homogenizer. Then, it was transferred into a centrifuge tube and centrifuged for 10 min (3000 r/s), and 0.5 ml of the supernatant was taken. After treatment, 25 *μ*l of the supernatant was injected for determination [14].

#### 3.2.3. Determination

In this paper, high-performance liquid chromatography was used to determine the chromatographic analysis conditions: I: 0.05 M sodium citrate-acetonitrile (volume ratio of 82/18) was used as the mobile phase, and the pH value was adjusted to 3.5 with triethylamine; the detection wavelength was 293 nm [15]. Chromatographic analysis condition II: PH4.2, 0.05 M sodium acetate, and methanol were prepared in the ratio of 32/68. A 0.45 *μ*l solvent filter was vacuum filtered before use, and the detection wavelength was 277 nm. The above two drugs were dried at 105°C for 2 hours and then weighed appropriately, and a standard solution was prepared by adding pH 7.4 phosphate buffer [16]. The peak area of levofloxacin was determined according to test condition I, the peak area of metronidazole was determined according to test condition II, and the standard curve equation was obtained with the measured peak area. Five samples of high, medium, and low concentrations were prepared according to the standard plasma preparation method to determine the peak area of each component. It is substituted into the respective regression equation to obtain the corresponding concentration finally [17].

The article "Mechanism of Anti-Inflammatory Drugs in the Early Treatment of Oral Gingival Mucosa and Soft Tissue Trauma" was retracted in 2023. Reasons: signs of a paper mill; compromised peer review; unreliable results or conclusions.

### 3.3. Data Processing

All measurement data were processed using Excel 2020 and SPSS 17.0 statistical software, and the data results were expressed as the mean ± standard deviation [18].

## 4. Role of Anti-Inflammatory Drugs in the Early Management of Gingival Mucosa and Soft Tissue Trauma

### 4.1. Animal Injury and Experimental Grouping

Twelve big-eared white rabbits were randomly divided into a control group and a medication group, 6 in each group. For each sample, the maxillary and mandibular incisor gingiva was studied, and 2 mm were removed from the gingiva with a scalpel. For the animals in the control group, the wounds were not treated; the animals in the medication group were administered 1 capsule per day, and the suture was delayed [19].

### 4.2. Observation Indicators and Methods

1. Wound healing
2. The wound healing of animals was observed at 12 h, 24 h, 3 d, 7 d, and 10 d
3. Changes in body temperature, respiratory rate, and heart rate
4. The changes in animal body temperature, respiratory rate, and heart rate were observed at 2 h, 6 h, 12 h, 24 h, 36 h, 3 d, and 7 d
5. Determination of intratissue pressure
6. At 2 h, 6 h, 12 h, 24 h, 36 h, 3 d, and 7 d, the pressure in the animal wound tissue was measured
7. Determination of tissue partial pressure of oxygen
8. At 2 h, 6 h, 12 h, 24 h, 36 h, 3 d, and 7 d, the partial pressure of oxygen in the wound tissue of animals was measured
9. Determination of IL-6 content
10. The content of IL-6 in animal wound tissue was measured at 12 h, 24 h, 3 d, 7 d, 10 d, 3 d, and 7 d
11. Determination of PGE2 content
12. The PGE2 content in animal wound tissue was measured at 12 h, 24 h, 3 d, 7 d, 10 d, 3 d, and 7 d [20]

## 5. Experimental Results and Discussion

### 5.1. Experimental Results of Drug Release Performance *In Vitro* and *In Vivo*

#### 5.1.1. Dissolution and Release of Drugs *In Vitro*

The release amounts of levofloxacin and metronidazole are shown in Table 1 and Figure 1.

The article "Mechanism of Anti-Inflammatory Drugs in the Early Treatment of Oral Gingival Mucosa and Soft Tissue Trauma" was retracted in 2023. Reasons: signs of a paper mill; compromised peer review; unreliable results or conclusions.

It can be seen from the data that the release of the two drugs *in vitro* is continuous and stable. The amount of the drug released gradually increased over time. At the 4th hour, the dissolution rate of levofloxacin was 27.83%. After the 24th hour, the dissolution rate reached 81.36%, indicating that the levofloxacin tablet had a good dissolution effect. The dissolution rate of metronidazole reached 34.58% in the 4th hour, and the dissolution rate was as high as 93.18% in the 24th hour, indicating that metronidazole tablets have a strong drug release ability. The *in vitro* release of the two drugs increased slowly from low to high, and the release was stable within 4–24 hours, and the drugs could be released stably and efficiently, which meets the release requirements of standard tablets, the requirements of this experiment, and the general drug metabolism law.

#### 5.1.2. Determination of Drug Distribution *In Vivo*

The maximum absorption wavelength of levofloxacin is 293 nm, and the levofloxacin in plasma (or tissue) is well separated, and the retention time is about 7.3 min, but metronidazole has no peak under analytical condition I. The chromatogram of levofloxacin is shown in Figure 2.

Metronidazole showed the maximum absorption at 277 nm wavelength. Under analytical condition II, levofloxacin and metronidazole were well separated, and the retention time of metronidazole was about 4.5 min. Peaks of other substances in the tablet can be seen at about 8.2 minutes. The chromatogram of metronidazole is shown in Figure 3.

#### 5.1.3. Linear Relationship

Each component drug in the tissue (plasma) has a good linear relationship, and the regression equation for levofloxacin is

(2) $$\begin{array}{c} Y=0.692X+0.077. \end{array}$$

The regression equation for metronidazole is

(3) $$\begin{array}{c} Y=0.0.476X+0.025. \end{array}$$

The correlation coefficient of levofloxacin was 0.9978, and the linear range was 0.02∼5.00 *μ*g/ml. The correlation coefficient of metronidazole was 0.9994, and the linear range was 0.03∼4.00 *μ*g/ml.

#### 5.1.4. Determination of Drug Concentration in the Sample

The drug distribution concentration in rabbits is shown in Table 2 and Figure 4.

As can be seen from the data, the concentrations of the two drugs in tissue and plasma increased first and then decreased with time. The concentrations of the two drugs were high in tissue and remained low in plasma. The drug concentration of levofloxacin in the tissue started at 6.54%, peaked at the 24th hour, and then decreased to 25.16% at the 36th hour. Plasma levofloxacin drug concentrations started at 0.07%, peaked at 24 hours, and then decreased to 1.25% at 36 hours. The concentration of metronidazole in the body is the same as that of levofloxacin. The drug concentration of metronidazole in the tissue started at 9.86%, and the drug concentration gradually increased with time, and the highest concentration was 92.61% at 24 hours and then began to decrease. The drug concentration of metronidazole in plasma started at 0.18%, and the drug concentration gradually increased with time, reaching the highest concentration at 24 hours at 7.49%, and then began to decrease. Comparing the drug concentrations of levofloxacin and metronidazole, it can be seen that the drug concentration of metronidazole is much higher than that of levofloxacin in both tissue and plasma, indicating that metronidazole has a better drug release capacity.

The article "Mechanism of Anti-Inflammatory Drugs in the Early Treatment of Oral Gingival Mucosa and Soft Tissue Trauma" was retracted in 2023. Reasons: signs of a paper mill; compromised peer review; unreliable results or conclusions.

The experimental results showed that the concentrations of the two drugs in the tissue were much higher than those in the plasma, and the retention time of the drugs in the tissue was long. The changing trend of the concentration at each point is relatively gentle, thus avoiding the adverse effects of local high concentrations on the wounded tissue and the whole body. Since the drug is released in a relatively stable manner within the cells, it not only has local anti-inflammatory effects but also reduces the toxic side effects in vivo.

### 5.2. The Role of Anti-Inflammatory Drugs in the Early Management of Gingival Mucosa and Soft Tissue Trauma

#### 5.2.1. Wound Healing

On the 12th hour, the injured gums in the control group were red, swollen, and bright, with viscous secretions exuding; the injured gums in the medication group were red and swollen, with fewer secretions.

On the 24th hour, tissue swelling was more obvious in the control group, with viscous secretions exuding, and bleeding was easy on light probing.

On the 3rd day, the gums in the control group were red, swollen, and bright, and no viscous secretions were seen. Some gums were covered with a white pseudomembrane, which was easy to bleed when probed.

On the 7th day, the gums of the control group were red and swollen, and the white pseudomembrane disappeared. No obvious granulation tissue was seen, and local exploration was bleeding. The redness and swelling of the gums in the medication group improved. No white pseudomembrane was seen, there was thin granulation tissue at the injury site, and the bleeding of the probe improved.

On the 10th day, the redness and swelling of the gingiva in the control group improved, there was no pseudomembrane, and a thin layer of granulation tissue was seen at the injury site, and there was no bleeding. In the medication group, gingival inflammation was improved, no white pseudomembrane was seen, and the granulation tissue at the injury site was thickened, and there was no bleeding.

The article "Mechanism of Anti-Inflammatory Drugs in the Early Treatment of Oral Gingival Mucosa and Soft Tissue Trauma" was retracted in 2023. Reasons: signs of a paper mill; compromised peer review; unreliable results or conclusions.

In general, the macroscopic observation showed that wound redness and swelling in the drug group were significantly improved. Compared with the wounds of the control animals at the same time point, tissue swelling was lighter, inflammation disappeared quickly, and wound recovery speed was faster.

#### 5.2.2. Changes in Body Temperature, Respiratory Rate, and Heart Rate

The changes in body temperature, respiratory rate, and heart rate of the two groups of animals after injury are shown in Figure 5.

The body temperature of animals before injury was 38.3°C. At the second hour, the body temperature of the animals in both groups decreased significantly. The body temperature of the control group dropped to 35.73°C, and the body temperature of the medication group dropped to 36.29°C. The body temperature of both groups of animals gradually increased over time. At the 12th hour, the temperature of the control group increased to 38.56°C, and the temperature of the medication group increased to 37.83°C. At the 36th hour, the body temperature of the two groups of animals reached the highest, the body temperature of the control group was 41.02°C, and the body temperature of the medication group was 39.25°C. Subsequently, the body temperature of the two groups of animals gradually decreased to the normal value. It can be seen from the data that although the changes in body temperature of the two groups of animals after injury are the same, compared with the control group, the body temperature of the medication group increases more slowly, indicating that anti-inflammatory drugs can effectively improve the body temperature changes caused by inflammation after injury.

The average respiratory rate of animals under anesthesia before injury was 49.37 breaths/min, and the respiratory rate decreased after injury. At 2 h, the respiratory rate of the control group was 32.36 times/min, and the respiratory rate of the medication group was 31.58 times/min. After 2 hours, the respiratory rate of the animals in the two groups increased significantly. At the 6th hour, the respiratory rate of the control group was 48.53 times/min, and the respiratory rate of the medication group was 45.32 times/min. After 2 hours, the respiratory rate of the animals in the two groups increased significantly. At the 6th hour, the respiratory rate of the control group was 48.53 times/min, and the respiratory rate of the medication group was 45.32 times/min. Then, over time, the body temperature of the animals in both groups increased slowly, with the control group rising faster and breathing more rapidly. At the 36th hour, the respiratory rate of the two groups of animals decreased until it decreased to the normal value. The heart rate of animals before the injury was 176.53 beats/min, and the heart rate of animals in both groups decreased significantly after injury. At the 2^nd^ hour, the heart rate of the control group was 141.87 beats/min, and the heart rate of the medication group was 130.68 beats/min. With the passage of time, the heart rate of animals in both groups gradually increased, and the heart rate of the control group increased more slowly. After the 12th hour, the heart rate of the control group and the medication group was significantly different. At the 12th hour, the heart rate of the control group was 187.29 beats/min, and the heart rate of the medication group was 196.32 beats/min. On the 36th hour, the heart rate of the control group was 197.85 beats/min, and the heart rate of the medication group was 215.37 beats/min. Then, the heart rate of the animals in both groups gradually decreased to the normal value. Overall, the heart rate was higher in the medication group.

The article "Mechanism of Anti-Inflammatory Drugs in the Early Treatment of Oral Gingival Mucosa and Soft Tissue Trauma" was retracted in 2023. Reasons: signs of a paper mill; compromised peer review; unreliable results or conclusions.

#### 5.2.3. Determination of Intratissue Pressure

Under the condition that the height is constant within 10 s before injury, the needle size and valve opening degree are the same, taking the number of liquid drops entering the muscle tissue as the standard, and the pressure change of the animal wound tissue was measured, as shown in Figure 6.

The preinjury animal tissue pressure was 1.00, and the postinjury tissue pressure increased significantly and gradually increased with time. At the second hour, the intratissue pressure of the control group was 1.19, and the intratissue pressure of the medication group was 1.15. With the passage of time, the intratissue pressure in the control group increased to 1.34 at the 12th hour, and the intratissue pressure in the medication group increased to 1.21. At the 36th hour, the intratissue pressure of the animals in the two groups rose to a high point, the intratissue pressure of the control group was 1.62, and the intratissue pressure of the medication group was 1.44, and then the intratissue pressure of the animals gradually decreased until normal. The observation data show that the pressure increase in the control group is larger, and the pressure change is more obvious, while the decrease speed is slower.

#### 5.2.4. Determination of Tissue Partial Pressure of Oxygen

Changes in oxygen partial pressure in animal wound tissues are shown in Figure 7.

The article "Mechanism of Anti-Inflammatory Drugs in the Early Treatment of Oral Gingival Mucosa and Soft Tissue Trauma" was retracted in 2023. Reasons: signs of a paper mill; compromised peer review; unreliable results or conclusions.

The partial pressure of oxygen in the tissues of the animals before injury was 31.22, and the partial pressure of oxygen in the tissues of the two groups of animals after injury showed a gradual downward trend. At the 2^nd^ hour, the oxygen partial pressure in the wound tissue of the two groups of animals was not much different; both were about 21. The tissue oxygen partial pressure in the treatment group increased briefly at the 6th hour and then continued to decrease. At the 12th hour, the tissue oxygen partial pressure in the control group was 18.08, and the tissue oxygen partial pressure in the medication group was 21.51. The difference in oxygen partial pressure between the two groups was large. At the 36^th^ hour, the tissue oxygen partial pressure in the control group was reduced to 14, and the tissue oxygen partial pressure in the medication group was reduced to 16.94. Subsequently, the partial pressure of oxygen in animal tissues gradually increased, and it was close to the preinjury level on the 7th day. It can be seen from the data that the decrease in tissue partial pressure of oxygen in the control group is greater, the rate of decline is faster, and the rate of recovery is slower, which is significantly different from that of the medication group.

#### 5.2.5. Determination of IL-6 Content

Figure 8 shows the changes in IL-6 content in wound tissue of the two groups of animals after injury.

The content of IL-6 in the tissue of animals before injury was 150.69 pg/g, and the content of IL-6 in the tissue of the wounded area of the two groups of animals after injury was significantly increased. At the 2^nd^ hour, the content of IL-6 in the tissues of the control group was 174.98 pg/g, and the content of IL-6 in the tissues of the treatment group was 186.24 pg/g. With the passage of time, the IL-6 content in the tissues of the two groups of animals gradually increased. At the 36th hour, the content of IL-6 in the tissues of the control group increased to 251.29 pg/g, and the content of IL-6 in the tissues of the treatment group increased to 213.57 pg/g and then gradually decreased. On the 7th day, the content of IL-6 in the tissue of the medication group reached the normal value, and the content of IL-6 in the tissue of the medication group was higher. Comparing the data of the two groups, it can be seen that the content of IL-6 in the control group increased rapidly, which was significantly higher than that in the medication group.

#### 5.2.6. Determination of PGE2 Content

The changes in PGE2 content in the wound tissue of the two groups of animals after injury are shown in Figure 9.

The article "Mechanism of Anti-Inflammatory Drugs in the Early Treatment of Oral Gingival Mucosa and Soft Tissue Trauma" was retracted in 2023. Reasons: signs of a paper mill; compromised peer review; unreliable results or conclusions.

The PGE2 content in the animal tissue before injury was 102.36 pg/g, and the PGE2 content in the wound tissue of the two groups of animals after injury was significantly increased. At the 2^nd^ h, the content of PGE2 in the tissues of the control group was 174.85 pg/g, and the content of PGE2 in the tissues of the treatment group was 158.23 pg/g. With the passage of time, the content of PGE2 in the tissues of the two groups of animals gradually increased. At the 36th hour, the content of PGE2 in the tissues of the control group increased to 249.81 pg/g, and the content of PGE2 in the tissues of the treatment group increased to 216.79 pg/g and then gradually decreased. On the 7th day, the content of PGE2 in the tissue of the medication group reached the normal value, while the content of PGE2 in the tissue of the medication group was higher. Comparing the data of the two groups, it can be seen that the content of PGE2 in the control group increased rapidly, which was significantly higher than that in the medication group.

### 5.3. Analysis of Experimental Results

The serum of trauma patients contains high levels of cytokines, such as IL-6 and TNF-*α*, and some other inflammatory mediators such as PGE2, leukotrienes, histamine, and others, which cause excessive inflammatory response in the body and cause damage to the body. Elevated levels of TNF-*α* in post-traumatic serum play an important role in causing many of the symptoms of SIRS (systemic inflammatory response syndrome). IL-6 is a cytokine mainly secreted by *T*, B cells and mononuclear macrophages, which can promote the activation and aggregation of neutrophils, and the concentration of IL-6 in serum can reflect the degree of tissue damage. As an inflammatory cytokine, PGE2 exists in inflammatory tissues and can act synergistically with inflammatory mediators such as bradykinin to aggravate the inflammatory response.

In this experiment, the inflammatory response of gingival soft tissue trauma was obvious, and the changing trend of the contents of PGE2, IL-6, and other mediators was consistent with the degree of tissue edema and partial pressure of oxygen. The surrounding tissue was significantly swollen, the oxygen partial pressure in the tissue was reduced, and there were more exudates. Body temperature and heart rate began to increase significantly 6 hours after the trauma, and it can be seen that excessive TNF-a and IL-6 lead to excessive inflammatory response. The results of this experiment have shown that anti-inflammatory drugs can significantly inhibit the content of PGE2 and IL-6 in the tissue after soft tissue injury and effectively inhibit the inflammatory response of soft tissue injury.

The article "Mechanism of Anti-Inflammatory Drugs in the Early Treatment of Oral Gingival Mucosa and Soft Tissue Trauma" was retracted in 2023. Reasons: signs of a paper mill; compromised peer review; unreliable results or conclusions.

## 6. Conclusion

In this paper, two anti-inflammatory drugs, levofloxacin and metronidazole, were selected. First, the release properties of the drugs *in vitro* and *in vivo* were measured. The results showed that both drugs had good release capabilities *in vitro* and *in vivo*. Then, the experiment of gingival wound treatment was carried out on white-eared rabbits, and various data of animals after injury were measured. The results showed that anti-inflammatory drugs can effectively reduce the inflammatory response. Compared with the control group, the physiological data of the animals in the administration group tended to stabilize faster, and the pressure in the wound tissue and the pressure change in the wound tissue were lower. The content of IL-6 and PGE2 in wound tissue increased more slowly, which was beneficial to the resolution of inflammation. Therefore, it can be determined that antistress drugs can promote wound healing by reducing the content of IL-6 and PGE2 in wound tissue.

## Figures and Tables

**Figure 1:** Drug *in vitro* dissolution.

**Figure 2:** Levofloxacin chromatogram.

**Figure 3:** Metronidazole chromatogram.

**Figure 4:** Drug distribution concentration in rabbits.

**Figure 5:** Changes in body temperature, respiratory rate, and heart rate after injury.

**Figure 6:** Animal wound tissue pressure.

**Figure 7:** Animal wound tissue partial pressure of oxygen.

**Figure 8:** Changes of IL-6 content in wound tissue of two groups of animals after injury.

**Figure 9:** Changes of TNF-a content in wound tissue of two groups of animals after injury.

**Table 1:** Drug *in vitro* dissolution.

Drug	Time after injury					
	4 h	8 h	12 h	16 h	20 h	24 h
Levofloxacin	27.83 ± 3.2	39.84 ± 2.8	50.37 ± 6.8	62.12 ± 2.4	70.56 ± 5.1	81.36 ± 3.2
Metronidazole	34.58 ± 6.2	49.76 ± 5.4	66.47 ± 3.5	75.48 ± 4.9	86.41 ± 5.7	93.18 ± 7.1

**Table 2:** Drug distribution concentration in rabbits.

Drug	Sample	Time after injury			
		6 h	12 h	24 h	36 h
Levofloxacin	Tissue	6.54 ± 1.21	32.83 ± 2.46	67.42 ± 4.58	25.16 ± 2.19
	Plasma	0.07 ± 0.04	1.43 ± 0.31	2.57 ± 0.98	1.25 ± 0.42

Metronidazole	Tissue	9.86 ± 1.74	57.92 ± 4.62	92.61 ± 8.66	41.39 ± 7.43
	Plasma	0.18 ± 0.08	4.24 ± 0.72	7.49 ± 1.17	3.58 ± 0.64

## Data Availability

The datasets generated during and/or analyzed during the current study are not publicly available due to sensitivity and data use agreement.
